The article "Construction of Rural Financial Organization Spatial Structure and Service Management Model Based on Deep Convolutional Neural Network" was retracted in 2023. Reasons: unreliable results or conclusions; concerns about the data; concerns about the peer review; concerns about the citations.

# Construction of Rural Financial Organization Spatial Structure and Service Management Model Based on Deep Convolutional Neural Network

**DOI:** 10.1155/2021/7974175

**Published:** 2021-07-06

**Authors:** Yan Liu

**Affiliations:** School of Economics and Management, Jilin Agricultural University, Changchun 130118, China

## Abstract

Local credit cooperatives have long played an important role in local financial services. It has made a significant contribution to agricultural production, farmers' incomes, and the economic development of rural areas. In particular, as a financial instrument serving farmers, microfinance management by local credit cooperatives plays a key role in pursuing profits and fulfilling social responsibility. It was therefore important to obtain effective instruments for combating poverty in rural areas from all walks of society. This paper first outlines the development of microfinance loans in Germany and other countries and describes the current situation and some of the challenges facing local credit cooperatives in financial management. Next, we present the basic concepts of data mining, describe the common methods and key techniques of data mining, analyze and compare the properties of the individual data, and show how the associated mining can actually be performed. Next, we will explain the basic model of microfinance for farmers and some risks in detail and analyze and evaluate the characteristics of these risks in the context of local credit cooperatives. As a result, this paper proposes an improved deep convolutional neural network. The optimized algorithm selects the optimal weight threshold value and different iteration times. The results are fewer errors, the results are closer to the correct data, and the efficiency is better than before. The algorithm is more efficient because errors have been greatly reduced and the time spent on them has been slightly reduced.

## 1. Introduction

In order to optimize the loan environment for farmers, better support the development of farmers, agriculture, and rural economy, strengthen the management of small credit loans to farmers, simplify the procedures of the loan process, standardize the actual operation behavior, and achieve sustainable business development, the People's Bank of China promulgated the Interim Measures for the Management of Small Credit Loans to Farmers by Rural Credit Societies as early as 1999 and required rural credit societies to open small credit loans to farmers according to local conditions [1]. This means that, in the past, small credit loans were mainly provided by organizations or NGOs [2]. This means that lending methods that used to be implemented mainly by organizations or nongovernmental institutions can now be carried out within the framework of the financial system, and through financial innovation, the central bank hopes to improve financial services for low- and middle-income groups of farmers who have guarantee capacity and lack collateral [3]. With the continuous promotion of the Central Bank, microcredit activities have been fully piloted and promoted and have been greatly developed. Rural credit unions are playing an increasingly important role in the microfinance arena [4]. Although microfinance for farmers has been well received by farmers and has played a positive role in the adjustment of rural economic structure and rural stability, farmers are a special group, agriculture is an inefficient and weak industry, and it relies on natural conditions. This uncertainty has led to frequent debt evasion and high nonperforming loan ratios for a long time, posing a high risk to the microfinance business [5, 6].

The article "Construction of Rural Financial Organization Spatial Structure and Service Management Model Based on Deep Convolutional Neural Network" was retracted in 2023. Reasons: unreliable results or conclusions; concerns about the data; concerns about the peer review; concerns about the citations.

There were many problems in the previous loan risk management, which brought huge losses to credit unions. With the massive accumulation of data and the improvement of the financial system, coupled with the fact that the restructuring of rural credit unions is in full swing, some of the original loan management systems are no longer able to meet the needs of the rapid development of credit union business and to properly manage and avoid loan risks [7]. Therefore, one of the pressing issues facing the banking industry is how to establish an effective credit risk assessment model to significantly reduce the credit risk of banks. At present, China's financial industry mainly uses manual rating of customer credit risk, which affects the accuracy and scientificity of the rating system to a certain extent because the manual assessment is mixed with many personal subjective factors. So is there a better way to solve this problem? The answer is yes. Data mining technology is an emerging discipline that can effectively solve these problems. If data mining technology is applied to credit evaluation models, it can alleviate some of the credit risk problems faced by the banking industry [8]. The use of computer technology, using data mining methods for classification and prediction, can be highly automated to organize and analyze the original data, and according to the predetermined induction and reasoning rules, the potential patterns can be mined and analyzed, as shown in Figure 1. The use of automatic classification implementation to classify customers' credit risk not only prevents the influence of human factors but also improves efficiency and speeds up processing. From the classification of commercial bank risk types, it believes that commercial bank risks include credit risk, liquidity risk, market risk, operational risk, policy risk, compliance risk, country risk, reputation risk, and strategic risk. Among them, compliance risk and legal risk are similar, and country risk, reputation risk, and strategic risk are almost absent or small in view of China's national conditions and the overall status of rural commercial banks [9]. From the relevant studies of rural commercial banks, Dong Numhui identified credit risk, liquidity risk, market risk, operational risk, and policy risk as the main risks of rural commercial banks and used the AHP method to evaluate the risks. The researchers concluded that the main risks of village banks are credit risk, policy risk, and operational risk and used qualitative analysis to analyze the risks and study the causes [10, 11]. The researchers used statistical analysis to construct a probit probability model to empirically analyze the sample data of farmers' loans provided by Hubei Rural Commercial Bank to explore the factors influencing credit risk [12]. They analyzed the causes of risk generation in rural commercial banks before merger and restructuring from five perspectives: credit risk, market risk, operational risk, policy risk, and reputation risk [13, 14].

The article "Construction of Rural Financial Organization Spatial Structure and Service Management Model Based on Deep Convolutional Neural Network" was retracted in 2023. Reasons: unreliable results or conclusions; concerns about the data; concerns about the peer review; concerns about the citations.

The researchers used the Copula function to integrate the three important risks of market, credit, and operation based on the data related to rural credit cooperatives, rural commercial banks, and rural cooperative banks to obtain the overall risk level of rural financial institutions. After summarizing the previous studies on credit risk and market risk of banks, researchers focus on the operational risk of small and medium-sized rural commercial banks and introduce the construction of an operational risk management system. Most of the literature in recent years has focused more on the study of credit risk and liquidity risk of rural commercial banks, followed by market risk, operational risk, and policy risk. Considering the availability of data, this study takes these five types of risks as the main part of rural commercial banks' risks. This paper first briefly describes the system development environment and tools, then implements the whole system through the implementation of system management module, customer information management module, loan application module, risk review and credit rating module, loan approval and lending review module, postloan management module, statistical query, and report module, and finally completes the system testing in terms of both functional testing and performance testing. Through the use of data mining technology and neural network technology, the whole paper implements the microcredit management system of agricultural and commercial banks, which achieves the intended objectives and effects of the system, enhances the microcredit business management ability of agricultural and commercial banks, and improves their working efficiency. The structure of the whole paper can be described as follows.

The article "Construction of Rural Financial Organization Spatial Structure and Service Management Model Based on Deep Convolutional Neural Network" was retracted in 2023. Reasons: unreliable results or conclusions; concerns about the data; concerns about the peer review; concerns about the citations.

In Section 2, we introduced the related work of microfinance and its applications in the related fields. In Section 3, this thesis introduced the deep convolutional neural network structure and main parameter settings. In Section 4, through the application research of intelligent devices, the realization of the functions of identity identification, environment perception, and data transmission of algorithm results is made faster.

## 2. Related Work

Microfinance was first researched and developed by Professor Yunus in 1976. After field research, Prof. Yunus found that the formal financial system was reluctant to lend to the poor, even with policy guidance, because of the harsh conditions. This led to a long period of unmet demand for financial resources from the poor. In the long run, without financial support, the poor will become poorer [15]. In order to change this situation, Professor Yunus established the Village Bank of Bangladesh by implementing microfinance. Practice shows that many poor people have been lifted out of poverty by the bank's provision of microcreditor loans to farmers. In 2006, Professor Yunus was awarded the Nobel Peace Prize in recognition of his efforts to promote economic and social development from the bottom of society [16].

Researchers believe that microfinance was created because the poor also need financial services. However, traditional formal financial institutions are very strict in the selection of their clients, especially for the trustee group, making it difficult for low-income people to access financial services. This contradicts with the strong demand of the low-income group. In order to reconcile this contradiction, microfinance was created as a financial and institutional innovation to build a bridge between the financial market and the poor, especially the credit market, so that the poor can have access to small-scale lending and financial market services [17]. This initiative not only alleviates poverty but also increases the potential for income generation and strongly contributes to the development of rural credit markets [18]. The researchers concluded that formal financial institutions have a significant advantage over other institutions in microfinance because of their wide distribution, faster market penetration, and experience in financial services. The researchers empirically investigated whether microfinance can eradicate poverty. The study confirmed the role of microcredit support in practice, showing that poor households supported by microcredit in the market are more risk-tolerant and have significantly higher welfare than poor households that do not receive microcredit [19].

The article "Construction of Rural Financial Organization Spatial Structure and Service Management Model Based on Deep Convolutional Neural Network" was retracted in 2023. Reasons: unreliable results or conclusions; concerns about the data; concerns about the peer review; concerns about the citations.

Researchers believe that the main constraints to the development of the rural economy are, first, the persistent weakness of farmers and, second, the persistent protectionism of the government. These have made the rural financial market extremely ineffective in terms of competitiveness. Other factors that researchers have identified as affecting the successful operation of microfinance are information asymmetry and collusion among farmers. These can affect the repayment rate of cobonded loans to some extent [20]. The researchers emphasize that the quality of the creditors themselves and the accuracy of the information collected from the farmers during the precredit survey are crucial to reducing the risk incidence. Further risk reduction can be achieved by limiting the amount of individual loans and overcollateralization, increasing risk provisions, carefully selecting the population, and making full use of credit ratings and incentives to repay loans. He reached these conclusions after investigating the current state of credit risk management in Latin American agricultural financial institutions [21]. The researchers took a shortcut and used a vector of high-dimensional data to abstractly describe the applicants [22, 23]. The benefit of this abstraction was the ability to use a nonlinear SVM to rate credit card applicants, with great success [24]. The researchers used LDA, decision trees, neural networks, and a model combining LDA and neural networks to conduct a credit risk assessment study on the same dataset separately, and the results showed that decision trees had the highest classification accuracy and linear discriminant analysis had the lowest accuracy of the four methods [25–27].

From the above research status, we can see that many scholars have made useful explorations in the study of microfinance for farmers. From the perspective of microcredit risk management to its effectiveness in poverty eradication, from commercial operation to development model, the scope of research is extremely broad. However, there are not many studies on microfinance credit risk management from the perspective of rural credit unions, and almost none of them are related to the internal credit risk control of rural credit unions.

## 3. Deep Convolutional Neural Network Structure and Main Parameter Settings

### 3.1. Neural Network Parameter Setting

*N*_2_ = 2*n*1 + 1; in this paper, the sample has 10 input parameters and 2 output parameters, so here 2*n* takes the value of 21; thus, the structure of the deep convolutional neural network is set as 10-21-2; that is, there are 10 nodes in the input layer, 21 nodes in the implicit layer, and 2 nodes in the output layer. Thus, the number of weights is 252 and the number of thresholds is 21 + 2 = 23. The number of parameters to be optimized in the ant colony algorithm is 252 + 23 = 275.

The article "Construction of Rural Financial Organization Spatial Structure and Service Management Model Based on Deep Convolutional Neural Network" was retracted in 2023. Reasons: unreliable results or conclusions; concerns about the data; concerns about the peer review; concerns about the citations.

A neural network is one that contains three layers (Figure 2). The convolution operation on the left is the input layer, the chaining operation on the right is the output layer, and pooling of nuclear is the middle layer (also called the hidden layer). In machine learning, deep convolutional neural network is a deep feedforward artificial neural network. If the number of implicit neurons is large enough, it can approximate any nonlinear function with finite discontinuity with arbitrary accuracy. In MATLAB, neural network toolbox requires that each column of the sample data matrix is a sample, so the input layer in this neural network has ten columns so the input layer is 10, the output layer has two columns so the output layer is 2, and the implied layer is 33.

Number of iterations: the minimum number of iterations is set to 200 for program testing, and the maximum number of iterations is set to 1000 for accuracy.

  Maximum number of iterations: set 1000.
  Pheromone volatility: 0.3%.
  Total pheromones: 1.0.
  Minimum error: 0.001.
  Actual error: 0.1.

After testing the data with MATLAB alone using the deep convolutional neural network algorithm, it can be concluded that when the number of iterations is set to 200, the error of the training sample is close to 0.11714 and stabilizes. When the number of iterations is set to 1000, the error of the training sample is close to 0.10494 and stabilizes. The results are shown in Figure 3. We use the modified deep convolutional neural network to classify the above data, respectively. It can be seen that the number of farmers with the actual result of “1” in the deep convolutional neural network algorithm before optimization is 966, and the number of farmers with the incorrect classification of “0” is 535. Among the 1499 individuals with attribute “0,” 1041 were correctly classified and 458 were incorrectly classified as “1,” and the correct classification rate of the algorithm before optimization was only 66.9%. For the same 3000 samples, the same analysis shows a significant improvement in the classification accuracy, reaching 91.3%.

### 3.2. Financial Organization of Convolutional Neural

Usually, the obtained sample data must be processed before it can be used in the network training process. Normalization is a way to simplify the computation by transforming a quantized expression, into a dimensionless expression, which becomes a scalar. To train the network using the ant colony algorithm, we need to quantize the input and output samples uniformly, generally uniformly as a real number between [0, 1]. In this paper, we normalize the output values in the interval according to the formula before learning.

The article "Construction of Rural Financial Organization Spatial Structure and Service Management Model Based on Deep Convolutional Neural Network" was retracted in 2023. Reasons: unreliable results or conclusions; concerns about the data; concerns about the peer review; concerns about the citations.

The main idea of the neural network algorithm is to construct a neural network through a series of computation and pruning process, where each middle node of the tree represents an attribute, the leaf node represents a classification category, and the branch goes to represent the value or range of the attribute. The most important thing in the tree construction process is the strategy of selecting decision attributes. The selection of attributes is based on a certain principle; that is, the attribute with the greatest information gain rate is selected as the candidate test decision attribute, and the information gain of the candidate attribute must be greater than or equal to the average of all attributes. Firstly, according to the principle of neural network algorithm, the expected information of the training sample data needs to be calculated. The expected information of this sample can be derived according to the algorithm's formula:

(1) $$\begin{array}{c} \text{MathExp}=-k\;\ln\left(\frac{A}{B}\right)-k^{\prime }\ln\left(\frac{A^{\prime }}{B^{\prime }}\right). \end{array}$$

Then calculate the entropy of each attribute, for example, the number of populations. The attribute has 3 category values, which can be derived from the formula

(2) $$\begin{array}{c} \text{Info}\left(M\right)=\frac{\text{MathExp}}{1+q}+i=\frac{-k\;\ln\left(A/B\right)-k^{\prime }\ln\left(A^{\prime }/B^{\prime }\right)+\left(1+q\right)i}{1+q}. \end{array}$$

According to the formula, the information gain of the number of farm household members is

(3) $$\begin{array}{c} S\left(\text{Info}\left(M\right)\right)=p{\left(\frac{\text{MathExp}}{1+q}+i\right)}^{l}=p{\left(\frac{-k\;\ln\left(A/B\right)-k^{\prime }\ln\left(A^{\prime }/B^{\prime }\right)+\left(1+q\right)i}{1+q}\right)}^{l}. \end{array}$$

Thus, the information gain rate of the population size is according to

(4) $$\begin{array}{c} G\left(\text{Info}\left(M\right)\right)=p^{\prime }{\left(\frac{\text{MathExp}}{1+q}+i\right)}^{l}=p^{\prime }{\left(\frac{-k\;\ln\left(A/B\right)-k^{\prime }\ln\left(A^{\prime }/B^{\prime }\right)+\left(1+q\right)i}{1+q}\right)}^{l}. \end{array}$$

According to the formula, the information gain of each attribute and the corresponding information gain rate are calculated, and then the neural network model is constructed by using the “top-down” recursive algorithm. Here, the classification attributes are selected based on the attributes with the largest information gain rate and the information gain that is not lower than the average of the information gain of all attributes as branch nodes. These factors also have a great influence on the credit union's risk assessment of small loans and can be used as an important basis for assessing the credit risk of borrowers.

The article "Construction of Rural Financial Organization Spatial Structure and Service Management Model Based on Deep Convolutional Neural Network" was retracted in 2023. Reasons: unreliable results or conclusions; concerns about the data; concerns about the peer review; concerns about the citations.

The above empirical analysis of the model by the neural network established for farmers has effectively illustrated the feasibility of this neural network model for micromanagement applications in rural financial management. Therefore, this paper constructs a compliant credit evaluation index system based on the model whose basic idea is that each attribute index value sets a different score according to the degree of importance of the farm household attributes identified by the neural network model. The size of the score is positively correlated with the influence of the attribute; that is, the greater the influence of the attribute is, the more important it is, and the corresponding score is higher. A score is then rated for each loaning farmer, and if the rated score reaches a multiboundary score, a loan is approved to be granted for financial management customer classification and loan risk management. The scoring model provides lenders with an objective tool to analyze the loan portfolio, making lender decisions faster and less costly. In addition to this, the scoring model is also applicable to assessing loan risk. The percentage scale quantifies the information provided by the farmer to obtain a certain value, but what credit rating does this value represent, for example, what does a score of “70” correspond to in practice? For this question, the next step is to determine the relationship between credit score and credit rating. To solve the problem of the relationship between credit score and credit rating of farmers, it is necessary to clarify the number and proportion of each credit rating in a random sample. The credit grades studied in this paper are mainly divided into four levels, namely, level 1, level 2, level 3, and level 4. After analyzing 4536 samples, the proportions of each level are 55.9%, 20.4%, 18.5%, and 5.2%, respectively. The 500 records from the test set were scored according to the evaluation model and analyzed according to the proportion of credit levels to obtain a rough credit rating scale, with 85–100 points as level 1, 70–85 points as level 2, 55–70 points as level 3, and 0–55 points as level 4.

The article "Construction of Rural Financial Organization Spatial Structure and Service Management Model Based on Deep Convolutional Neural Network" was retracted in 2023. Reasons: unreliable results or conclusions; concerns about the data; concerns about the peer review; concerns about the citations.

### 3.3. Management Model Risk Assessment

As the rural financial management business continues to expand and the decision-making requirements continue to increase, the traditional financial management system is becoming increasingly overwhelmed and reveals many shortcomings. Therefore, it is necessary to design and develop a financial management system with risk management capability and decision support. Due to the booming development of the Internet, more and more data and information need to be processed, which requires that it must also achieve the following goals and functions: First, the networking of financial management to facilitate data collection as well as knowledge sharing. Second, the scientificization of financial management decision-making. The system should have the ability to assist, regulate, control, and constrain financial management decision-making behavior and be able to rely on data mining tools for data discovery and analysis in order to make more scientific decisions and reduce prelending risks. Third, the refinement of financial management. The system will establish the refinement management of prelending forecast and postlending inspection and is able to penetrate the management level into each life cycle of financial management business. Fourth, the immediacy of financial management asset supervision. This means that the system needs to have a financial management risk warning function and be able to rely on the network to provide timely supervision and management of the institution's financial management assets. Relying on the data mining system to analyze and discriminate risk events and risky customers, it automatically identifies financial management risks that will occur and alerts financial management managers for early warning. Fifth, data sharing and knowledge sharing with other systems within the bank which is realized. Through the standardized interface developed by the institution, other systems are accessed according to the unified interface provided by the financial management system, reducing the workload of inputting data from the financial management system and other business management systems and ensuring the consistency of the shared data.

The main functions of the financial management system include the following parts: it can manage the financial management customers, daily loans, and loan risks of rural credit cooperatives and provide scientific decision support, so as to realize the standardization, science, and automation of financial management and effectively prevent or solve various risks in financial management business. It can be roughly divided into the following functional modules: data mining, customer management, risk management, financial management business, and system maintenance. The functional modules of the financial management system are shown in Figure 4.

The article "Construction of Rural Financial Organization Spatial Structure and Service Management Model Based on Deep Convolutional Neural Network" was retracted in 2023. Reasons: unreliable results or conclusions; concerns about the data; concerns about the peer review; concerns about the citations.

The first step in data mining is to figure out the substantive purpose of mining and define the business need or problem. As shown in Figure 5, the relationship between risk level and financial management income shows a significant positive correlation. The functional requirement of management model risk assessment is to analyze the level of financial management risk of farmers based on personal related information, credit reports, applications, and households of farmers using mathematical tools to get quantitative results and then use the results as the basis of whether to lend or not to make financial management decisions scientifically and automatically.

Data quality involves many factors, including accuracy, completeness, consistency, timeliness, credibility, and interpretability. Firstly, it is important to remove those sample data that are not relevant to the experiment, that is, data that are not relevant to the credit risk assessment of farmers' microfinance. The sample data collected are considered to be real user data from the credit union database, relevant to the modeling, and carefully prepared and therefore do not need to be removed. The next step is to remove attributes from the sample data that are not relevant to modeling. There are various pieces of user attribute information in the database of agricultural credit unions, but most of them are not related to the credit assessment of farmers' small loans, such as user name, loan institution name, loan number, home address, communication method, loan document number, loan account number, account manager, and main account manager. In the data preparation part, the redundant attributes were removed during the query process of the sample data. At the same time, it is also necessary to remove those redundant attributes. The so-called redundancy is that one attribute can be inferred from another attribute, or two attributes have the same meaning, but they are expressed in different ways. The mining model is independently influenced by each attribute value, and the presence of redundant attribute values can have an impact on the accuracy of the classification and prediction model. It is difficult to determine which attributes are redundant or irrelevant in the data preprocessing process, and Weka, a number mining software, is used to analyze the attribute values during the experiment.

The sample data come from multiple databases and there is variability in their data formats. In order to conduct the experiment properly, necessary conversions must be performed on some of the nonstandard sample data, such as the conversion of nominal values to numerical types and normalization operations of the data. The data cleaning process is complicated, and a reasonable data cleaning strategy must be developed based on the actual situation of the sample data and after data analysis. The data cleaning process of this experiment mainly applies manual screening in the form of sample information processing, and the data with null values, obvious errors, and noise are corrected using different strategies to make them meet the requirements of mining modeling. For example, for null data, the average value can be used to fill the method. After the data cleaning process, the sample data become more clean and tidy, which provides a strong data basis for the training and validation of the mining model. After a series of preprocessing of the sample data, a training sample set suitable for the data mining task is extracted, as shown in Figure 6. This training sample set consists of 80 records, each consisting of the following fields: population, marital status, labor force, net worth, total household property, credit union shares, net income, overall rating, and repayment history, with each attribute taking values normalized to good customer, medium customer, and bad customer.

The article "Construction of Rural Financial Organization Spatial Structure and Service Management Model Based on Deep Convolutional Neural Network" was retracted in 2023. Reasons: unreliable results or conclusions; concerns about the data; concerns about the peer review; concerns about the citations.

## 4. Comparison and Analysis of Algorithm Results

From the data input and the result output, it can be concluded that the algorithm optimization of the deep convolutional neural network is more effective and the error is smaller to some extent. It can be seen that the overall accuracy of the algorithm is improved significantly after the optimization of the weights and thresholds of the deep convolutional neural network. The sim function in the MATLAB toolbox is used to run the Simulink model to simulate the values of the input condition variables, the norm function in the toolbox is called to calculate the norm of the test data matrix through the program to obtain the sample simulation error, and thus, the comparison shows that the algorithm has a lower error, shorter computation time, and higher efficiency. The ROC curves are plotted with the true positive rate as the vertical coordinate and the false positive rate as the horizontal coordinate according to the different dichotomous classification methods, and the closer the ROC curve is to the upper left corner, the higher the accuracy of the test is. The point of the ROC curve closest to the upper left corner is the best threshold with the least number of errors and the lowest total number of false positives and false negatives. The area under the ROC curve has values between 1.0 and 0.5. An area under the curve greater than 0.5 indicates a better diagnosis. The area under the curve had low accuracy at 0.5 to 0.7, some accuracy at 0.7 to 0.9, and high accuracy at AUC above 0.9. As to the accuracy of the approach, with the help of the optimization of the weights and thresholds, this algorithm shows that a much lower error fluctuates to 0.05%. The ROC curves were obtained by comparing the classification results obtained from such models before improvement with the correct results through SPSS software, as shown in Figure 7; the area under the curve is equal to 0.827 > 0.7.

The article "Construction of Rural Financial Organization Spatial Structure and Service Management Model Based on Deep Convolutional Neural Network" was retracted in 2023. Reasons: unreliable results or conclusions; concerns about the data; concerns about the peer review; concerns about the citations.

This marked red point (0.075, 0.096) has high sensitivity, high specificity, and the least number of false negatives and false positives. The ROC curve was obtained by comparing the classification results obtained from this improved model with the correct results through SPSS software, and the area under the curve is equal to 0.877 > 0.7 as shown in Figure 8. The red dots (0.107, 0.861) are marked with higher sensitivity, higher specificity, and the least false negatives and false positives. By comparison, we can find that the improved classification model is better than the previous model in terms of classification effect. In today's technological era of rapid information development, the development of data mining technology has also entered a new peak. It has gradually become the focus of our current database and related artificial intelligence fields to be studied. In terms of the development process of neural networks, theoretical research is often at the forefront and sometimes beyond the practical use stage. Although theoretical research and practical applications can complement each other, practical needs are always the main driving force of technological development. At present, there are many practical applications of neural networks, such as intelligent control, pattern recognition, and robot control. It can be seen that making full use of neural network algorithms to process the required data can increase its application in real life.

In neural networks, the weights are automatically generated; initially, each weight is generated by a random number function with values ranging between [−1, 1], then the neural network is trained according to the training data, and during the training process, the neural network automatically adjusts the weights according to the output error to achieve the output requirements. In neural networks, the threshold value, as a critical value, is the lowest or highest value that an effect can produce. Since neural networks mimic neurons in the brain, a neuron is only stimulated when an external stimulus reaches a certain threshold value, affecting the next neuron. The selection of weights and thresholds in the neural network algorithm is random. The weights and thresholds are continuously updated as the number of algorithm evolutions increases. This random selection process usually leads to an increase in the number of iterations of the algorithm, an increase in the running time, and a decrease in the optimization accuracy, which affects the execution efficiency of the algorithm. From the data input and result output, it can be concluded that the algorithm optimization of the deep convolutional neural network is more effective and the error is smaller to a certain extent. The process of solving the optimal solution is equivalent to finding a set of optimal weights and threshold combinations. To overcome the problem of random selection of weights and thresholds, in this paper, we use the global optimization capability of the ant colony algorithm to optimize the initial selection and thresholds of the deep convolutional neural network in order to improve the construction efficiency and prediction accuracy of the neural network model. Then, the optimized weights and thresholds are brought into the corresponding algorithm to derive the error-optimal prediction results.

The article "Construction of Rural Financial Organization Spatial Structure and Service Management Model Based on Deep Convolutional Neural Network" was retracted in 2023. Reasons: unreliable results or conclusions; concerns about the data; concerns about the peer review; concerns about the citations.

Therefore, it is necessary to design and develop a financial management system with risk management capability and decision support. Due to the booming development of the Internet, more and more data and information need to be processed, which requires that it must also achieve the following goals and functions: First, the networking of financial management to facilitate data collection as well as knowledge sharing. Second, the scientificization of financial management decision-making. The system should have the ability to assist, regulate, control, and constrain financial management decision-making behavior and be able to rely on data mining tools for data discovery and analysis in order to make more scientific decisions and reduce prelending risks. Third, the refinement of financial management.

## 5. Conclusion

Combining deep convolutional neural network algorithms using rural credit union farmer credit rating and data mining technology can provide good technology to rural credit unions to support the control of potential loan risks of farmers. In this paper, we analyze some applications and feasibility of data mining technology in improving the financial management of rural credit unions based on the actual situation of rural credit unions, combined with previous data mining research results. Then based on rural credit unions, it analyzes in detail the problems of data warehouse construction and data mining models for loan management, proposes relevant design models and specific implementation methods with suitable financial management systems according to the characteristics of rural credit unions, and realizes an intelligent auxiliary analysis system for financial management risks of small farmers. This paper proposes how to design the financial management system based on data mining and the specific implementation method. The system mainly includes the following functional modules: financial management business, customer management, data mining module, and financial management risk management. The core functions of the designed system are the monitoring and management of the whole process of credit and financial management of rural credit cooperatives, the realistic and effective customer management of lending business, data mining management, and financial management risk management. It aims to realize the effective embedding of data mining function and financial management, as well as decision support, eventually realize the scientific, standardization, and automation of financial management, and effectively prevent or solve financial management business risks.

The article "Construction of Rural Financial Organization Spatial Structure and Service Management Model Based on Deep Convolutional Neural Network" was retracted in 2023. Reasons: unreliable results or conclusions; concerns about the data; concerns about the peer review; concerns about the citations.

## Figures and Tables

**Figure 1:** Credit evaluation model based on deep convolutional neural network data mining.

**Figure 2:** Deep convolutional neural network at multiple iterations.

**Figure 3:** Error analysis of deep convolutional neural network at multiple iterations.

**Figure 4:** Spatial structure of financial management organization.

**Figure 5:** Relationship between risk level and financial management income.

**Figure 6:** Credit assessment analysis by attribute.

**Figure 7:** Cross-tabulation of prediction and sample levels.

**Figure 8:** Comparison of the accuracy of the models.

## Data Availability

The data used to support the findings of this study are available from the author upon request.
